# Development and Verification of Prognostic Nomogram for Penile Cancer Based on the SEER Database

**DOI:** 10.1155/2022/8752388

**Published:** 2022-04-04

**Authors:** Yon-Bo Chen, Ying-Wen Liu, Liang Gao, Liang-You Tang, Jiang Guo, Yu-Chang Tian, Ping-Hong You

**Affiliations:** ^1^Department of Urology, People's Hospital of Deyang City, China 173# Northern Taishan Road, Deyang, CN 618000; ^2^Department of Laboratory, People's Hospital of Deyang City, China 173# Northern Taishan Road, Deyang, CN 618000; ^3^Department of Urology, The Second Affiliated Hospital of Chongqing Medical University, China 74# Linjiang Road, Chongqing, CN 400010

## Abstract

**Aim:**

We aimed to establish a prognostic nomogram for penile cancer (PC) patients based on the Surveillance, Epidemiology, and End Results Program (SEER) database.

**Methods:**

Data from 1643 patients between 2010 and 2015 were downloaded and extracted from the SEER database. They were randomly divided into the development group (70%) and the verification group (30%), and then, univariate and multivariate Cox proportional hazards regression, respectively, was used to explore the possible risk factors of PC. The factors significantly related to overall survival (OS) and cancer-specific survival (CSS) were used to establish the nomogram, which was assessed via the concordance index (C-index), receiver operating characteristic (ROC) curve, and calibration curve. An internal validation was conducted to test the accuracy and effectiveness of the nomogram. Kaplan–Meier calculation was used to predict the further OS and CSS status of these patients.

**Results:**

On multivariate Cox proportional hazards regression, the independent prognostic risk factors associated with OS were age, race, marital status, N/M stage, surgery, surgery of lymph nodes, and histologic type, with a moderate C-index of 0.737 (95% confidence interval (CI): 0.713–0.760) and 0.766 (95% CI: 0.731–0.801) in the development and verification groups, respectively. The areas under the ROC (AUC) of 3- and 5-year OS were 0.749 and 0.770, respectively. While marital status, N/M stage, surgery, surgery of lymph nodes, and histologic type were significantly linked to PC patients' CSS, which have better C-index of 0.802 (95% confidence interval (CI): 0.771–0.833) and 0.82 (95% CI: 0.775–0.865) in the development and verification groups, and the AUC of 3- and 5-year CSS were 0.766 and 0.787. Both of the survival calibration curves of 3- and 5-year OS and CSS brought out a high consistency.

**Conclusion:**

Our study produced a satisfactory nomogram revealing the survival of PC patients, which could be helpful for clinicians to assess the situation of PC patients and to implement further treatment.

## 1. Introduction

Although its incidence increased slightly in some areas in recent years, penile cancer (PC) is still a relatively rare malignancy in developed countries [1–3]. Multiple etiologies have been suggested to contribute to the development of this disease, such as human papillomavirus (HPV) infection, phimosis, lichen sclerosis, smoking, condylomata acuminata, sexual problems, and chronic inflammation, among others [4–10].

Because of its high mortality, a clinical model for predicting the prognosis of PC patients is necessary [11]. Although the TNM stage and pathological classification systems from the 8th American Joint Committee on Cancer (AJCC) and the Union for International Cancer Control were widely used to predict the survival of PC patients [12, 13], a lot of limitations existed.

As we know, the patient's prognosis is individual. And multiple factors other than TNM staging would have independently affected patients' prognosis, including age, race, marital status, information of surgery, count and density of examined lymph node, and histologic type [14, 15]. The nomogram can quantify and analyze these factors more comprehensively than TNM staging system and finally get a more specific value of event probabilities [16]. It can help clinicians and patients to obtain reliable prognostic information more individual, reliable, and convenient [17, 18].

It should be noted that the application of nomogram is limited by the established population, and it must be carefully cautioned when it is applied to different populations. However, the bias can be reduced by increasing the sample size. The Surveillance, Epidemiology, and End Results Program (SEER) database had collected detailed information on PC patients from multicenter in America, which allowed us to build a reliable prognostic nomogram.

## 2. Methods

After registering an account and signing a Data Agreement on the SEER database website, we were authorized to download all the data of PC patients using the SEER ∗ Stat version 8.3.5 software. All available data on the patients' age, race, marital status, TNM stage (AJCC 7th standard 2010+), tumor primary site, surgery, surgery of lymph nodes, radiation, chemotherapy, histologic type, survival time, cancer-cause death, and live status were collected. Cases with unknown, undefined, or missing data were excluded. Patients' prognosis was mainly evaluated by the outcome of overall survival (OS) and cancer-specific survival (CSS). The “caret” package of the R version 3.6.0 software was utilized to randomize the patients into the development group (70%) and the verification group (30%). Notably, in our study, the patients' histologic type was limited to squamous cell neoplasms based on the 3rd Edition (ICD-O-3) (805-808). Patients with a follow-up less than 1 month were removed. Patients whose race is not black or white are described as “others,” and patients who are divorced, separated, widowed, and unmarried but have a domestic partner are considered as “single.”

The R version 3.6.0 software with the “foreign,” “survival,” “survminer,” and “rms” packages was used in all statistical analyses, and a *P* value of < 0.05 was regarded to be statistically significant. Every parameter was first analyzed using the univariate and multivariate Cox proportional hazards regression model to calculate hazard ratio and 95% confidence interval (CI). Then, possible risk factors linked to OS and CSS were identified. Finally, on the basis of those independent prognostic risk factors, the prognostic nomogram was developed to predict patients' further OS and CSS.

The concordance index (C-index), area under the receiver operating characteristic curve (AUC), and calibration curves of 3- and 5-year OS and CSS were calculated to verify the accuracy of the nomogram. Higher C-index and more AUC meant higher quality. We set up as many as possible bootstraps with 1000 resamples to ensure the precision of 3- and 5-year calibrations in comparing the predicted and observed OS and CSS. Furthermore, the Kaplan–Meier analysis was also used to demonstrate patients' possible OS and CSS.

## 3. Results

According to the screening criteria, 1943 males between 2010 and 2015 were involved in our study, from which 300 patients were excluded because of incomplete clinical information. Eventually, 1643 patients were included and then randomly divided into the development group (1151 patients) and the validation group (492 patients). The characteristics of these patients are summarized in Table 1.

In the development group, the median follow-up time was 42 (95% CI: 40–46) months, whereas the median OS was 66 (95% CI: 57–NA) months, and the median CSS was unavailable (Figures 1(a) and 1(b)). The univariate and multivariate COX regression analyses were carried out to predict patients' OS and CSS and identify the independent prognostic factors of PC (Tables 2 and 3). On univariate Cox proportional hazards regression, age, marital status, TNM stage, surgery, radiation, chemotherapy, and histologic type were all significantly related to the OS of PC patients, while marital status, TNM stage, primary site, surgery, surgery of lymph nodes, radiation, chemotherapy, and histologic type were associated to CSS. On multivariate Cox regression, the prognostic factors related to OS and CSS that were strongly independent included marital status, N/M stage, surgery, surgery of lymph nodes, and histologic type. Age and race could only affect patients' OS independently. Additionally, insignificant correlation of OS and CSS was found for T stage, tumor primary site radiation, and chemotherapy.

The prognostic nomogram involving all risk factors might be related to patients' OS or CSS based on the data of the development group is shown in Figures 2(a) and 2(b). Corresponding scores were assigned to each factor, and the sum of scores reflected the 3- and 5-year OS and CSS and mortality of patients. The C-index of the nomogram model for predicting the OS based on the development group was 0.737 (95% CI: 0.713–0.760), whereas that based on the verification group was significantly superior, with a value of 0.766 (95% CI: 0.731–0.801). Nomogram for predicting CSS showed better reliability and stability, with the C-index of 0.802 (95% confidence interval (CI): 0.771–0.833) and 0.82 (95% CI: 0.775–0.865) in the development and verification groups. The AUC of 3-year OS and CSS were 0.749 and 0.766 and of 5-year OS and CSS were 0.770 and 0.787 in the development group (Figures 3(a) and 3(b)), respectively, which indicated the reliability of these two nomograms. Both of the 3- and 5-year calibration curves predicted that the OS and CSS of the development group also showed satisfactory consistency between the observed and predicted outcomes (Figures 3(c) and 3(d)).

More intuitional differences of OS and CSS were shown on Kaplan–Meier analyses. The “coxph” package was used to build the proportional-risk model. After comparing their median risk, patients were divided into high- and low-risk groups, from which the high-risk group had both lower 3 years OS (43.7%, 95% CI: 39.5%–48.4%) and CSS (69.6%, 95% CI: 65.2%–74.3%), as well as had worse 5 years OS (31.1%, 95% CI: 26.4%–36.5%) and CSS (65.9%, 95% CI: 60.8%–71.5%) (*P* < 0.0001) (Figures 3(e) and 3(f)). Furthermore, patients aged >80 and 70–79 years had significantly lower OS than younger patients had (*P* < 0.0001) (Figure 4(a)), while younger patients had not an obvious advantage in CSS (Figure 4(b)). Marital status also seemed to affect the survival, as single patients were found to have a lower OS than others (*P* < 0.0001), and patients who never married unexpectedly got a worse CSS (*P* = 0.025); married patients had significant superiority over others in OS and CSS (Figures 4(c) and 4(d)). Although patients with more than four lymph nodes removed had a slight but insignificant advantage in OS, lymph node surgery did not contribute significant benefit (*P* = 0.059) (Figure 4(e)) and was even associated with poorer CSS (*P* < 0.0001) (Figure 4(f)). The impact of pathological differences on prognosis was obvious, in which verrucous and papillary carcinoma had significantly better OS and CSS (Figures 4(g) and 4(h)). No significant difference in OS and CSS was found among patients of different races or tumor primary sites; nevertheless, it seemed that patients would get a better survival when the primary tumor was located at the prepuce (Figures 4(i)–4(l)). However, significant differences of OS and CSS in Kaplan–Meier curves were also observed in the TNM stage, surgery, radiation, and chemotherapy (Figures 5(a)–5(l)). The OS and CSS of patients receiving radical surgery, radiotherapy, and chemotherapy did not significantly improve either, although patients who received preoperative radiotherapy seemed to get a better CSS.

C-index, AUC, and calibration curves were used to evaluate the accuracy of the two nomograms. The verification group had a C-index of 0.766 (95% CI: 0.731–0.801) and 0.82 (95% CI: 0.775–0.865) when predicting the OS and CSS, respectively, which were both higher and better than those of the development group. Meanwhile, the AUC of 3-year OS and CSS in the validation group were 0.754 and 0.771 and of 5-year OS and CSS were 0.723 and 0.756 (Figures 6(a) and 6(b)). The observed-predicted calibration curve at 3 and 5 years also showed similar results (Figures 6(c) and 6(d)). All of these results demonstrate the accuracy of these nomograms.

## 4. Discussion

Although patients have some differences in hygienic, social, and religious practice [19], PC, mostly squamous cell carcinoma [20], has been a rare disease in the past decades [21–23]. In most developed areas, the incidence of PC has been gradually decreasing [24, 25]. However, because of the uncommon clinical cases and lack of reliable prognostic tools, clinicians seemed to have limited methods for understanding and predicting the prognosis of PC.

As a tool for predicting patients' prognosis, the nomogram is widely used in oncology, such as in bladder, prostatic, and breast cancer [26–28]. It can provide a more individualized prognostic assessment for patients by combining various prognostic risk factors which have been widely recognized [29]. Our prognostic nomogram was based on the SEER database, which includes the detailed information of approximately 34.6% of the U.S. population [30].

In our study, elderly patients, especially those older than 80 years, would have a significantly lower 3-year (38.9%, 95% CI: 32.9%–42.1%) and 5-year (22.7%, 95% CI: 16.8%–30.8%) overall survival (*P* < 0.0001). Simultaneously, multivariate Cox analyses also revealed the risk of advanced age; these patients were weighted with more points than others in the nomogram. Furthermore, the Kaplan–Meier curve of age showed only slight differences in OS among all groups younger than 70 years (597/1151 of the development group). These findings suggest that elder age may be an independent risk factor for the prognosis of PC patients, which is consistent with most studies [23]. However, the difference in age in our study did not affect patients' CSS, as reported in the study of Shao et al. [31].

According to a study that included 5412 patients from the SEER who suffered penile squamous cell carcinoma between 1998 and 2011 by Sharma et al., black males who suffered from PC would have a worse OS. However, they excluded all patients in the M1 stage and included only 183 black patients, most of whom were diagnosed with a higher T stage of disease, lacked private insurance, and had lower median income [32]. Similarly, Slopnick et al. declared that African–American (AA) PC patients probably had a higher risk of death than white patients. Compared to white patients, surgical treatment was significantly delayed in AA patients. Meanwhile, a higher incidence of medical comorbidities such as heart disease, hypertension, and diabetes might also reduce their OS [33]. In our study, the white race was also an independent prognostic factor of OS but not CSS based on the Cox regression, but Kaplan–Meier curve analyses demonstrated that white patients only had a slight advantage in the long-term OS compared to black and other races. Thus, it may be worthwhile to explore higher mortality rates among different areas rather than among different races.

We also focused on marital status in our study. Cox regression analyses revealed that married status independently affects OS and CSS; married males with PC had better survival than single or unmarried patients, which might be related to their relatively fixed sexual partners or regular and clean sexual practices. Both intentional and unintentional examinations by the married male or his spouse before and after intercourse could also allow for the detection of penile abnormalities in the early stage. Unexpectedly, although the average age of unmarried men was younger, their survival still had no sufficient advantages, even worse than the single patients in CSS.

Furthermore, the results of Cox regression analyses suggested the importance of the cancer stage in the prognostic evaluation of patients. However, this seemed that the T stage did not show sufficient prognostic value in the multivariate Cox regression, which was consistent with the result from Gao et al. [14]. In the K-M analysis, the T stage was obviously related to patients' survival. Wu et al. included 234 patients from Sun Yat-Sen University Cancer Hospital and declared that the pathological T stage was an independent risk factor of lymph node metastases [34]. Similar to most studies, lymph node involvement and distant metastasis were found to be independent risk factors for prognosis [35]. Notably, our results also showed that the absence of significantly enlarged lymph nodes in the groin was very important for prognosis.

A different tumor primary site would not affect the prognosis of PC patients; clinicians should thus decide on the appropriate surgical method based more on the stage of the tumor to preserve the patients' sexual ability and improve sexual satisfaction. Expectedly, patients who underwent surgery showed generally better CSS; particularly, the therapeutic effects of electrocautery, fulguration, cryosurgery, and laser ablation were worthy of recognition. However, the prognosis of patients after radical surgery did not improve significantly. They generally had a worse TNM stage; this might be the cause of poor prognosis. But there may be a statistical bias because only a few patients (0.2%) underwent debulking surgery. Nevertheless, considering the integrity of the data, we still retained this in our calculation.

The recent guidelines on PC from the European Association of Urology strongly affirmed the prognostic importance of the number of positive lymph nodes found on physical examination and pathological biopsy. The OS of patients with three or more inguinal lymph nodes would drop sharply to below 60% [36, 37]. However, in our study, the K-M curve showed insignificant difference in OS between patients with different numbers of lymph nodes surgically removed, and patients whose lymph nodes were not removed had a better CSS. Hakenberg et al. claimed that 25% of patients might have micrometastases; even if they did not have obvious swollen inguinal lymph nodes, they might have early metastasized [38]. Thus, surgeons should prospectively focus on sentinel lymph node biopsy or dynamic sentinel lymph node biopsy to determine lymph node metastasis as accurately as possible, rather than simply predicting the prognosis and formulating treatment plans based on the number of enlarged lymph nodes found on physical examination or removed in surgery [39, 40].

Most studies have found that adjuvant chemotherapy could improve the disease-free survival rate and median survival of PC patients with positive lymph nodes after radical inguinal lymph node dissection [41, 42], and this might also reduce their clinical stage [43, 44]. However, our results showed that chemotherapy was not an independent prognostic risk factor. In the development group, patients receiving chemotherapy (141 patients) had significantly wider lymph node infiltration on average (stage N2: 37 patients, stage N3: 48 patients), which was also considered to be a high-risk factor for recurrence after chemotherapy [45]. Since the data were unclear about the specific chemotherapy regimens given, we were conservative about this result. Patients who received radiotherapy either before or after surgery did not have significant benefits and even had worse survival. Patients who received preoperative radiotherapy seemed to get a better CSS, but a bias might be caused by limited patient number (2/1151). Radiation therapy would increase the difficulty and the risk of complications in the dissection of inguinal positive lymph nodes and resection of the primary tumor. Some studies also claimed that radiation therapy cannot significantly prolong the OS of PC patients [46, 47]. Our study also found that the pathological characteristic of patients was an important factor of prognosis, among which verrucous carcinoma, verrucous papilloma, squamous cell papilloma, and papillary squamous cell carcinoma (ICD-O-3: 8051, 8052) would be protective. However, Bowen disease, basaloid squamous cell carcinoma and squamous cell carcinoma, and clear cell type (ICD-O-3: 8081, 8083, 8084) were the opposite, and the squamous cell carcinoma was intermediate, which was consistent with most studies [38].

Some limitations in our study must be taken into consideration. First, the SEER database was a retrospective resource library including patients from USA over a long period of time. Most of these patients were white, which might have introduced a bias and limited its application. Second, data about habits, customs (especially for sexual activity), HPV infection, average income, religion, smoking, education, Charlson comorbidity index, complications, and other information were not available in the SEER database, which could also affect the quality of our results. Finally, no additional data about PC patients from other sources or institutions could be used for external verification, which might have caused a selection bias.

## 5. Conclusions

Our results demonstrated that our nomogram model is feasible and reliable. This could be helpful for clinicians to evaluate the prognosis of PC patients faster and more accurately. However, because of the limitations in our study, more prospective studies are required to verify the accuracy of this nomogram.

## Figures and Tables

**Figure 1:** The Kaplan-Meier (KM) curves for predicting the OS (a) and CSS (b) of PC patients in the development group.

**Figure 2:** Prognostic nomograms for predicting the OS (a) and CSS (b) probability.

**Figure 3:** 3- and 5-year receiver operating characteristic curves (ROC) of the development group when predicting the OS (a) and CSS (b); 3- and 5-year calibration curves of the development group when predicting the OS (c) and CSS (d); Kaplan-Meier curves of OS and CSS based on risk_level (e, f).

**Figure 4:** Kaplan-Meier curves of OS and CSS based on age (a, b), marital status (c, d), surgery_LN (e, f), histologic type (g, h), race (i, j), and primary site (k, l).

**Figure 5:** Kaplan-Meier curves of OS and CSS based on stage_T (a, b), stage_N (c, d), stage_M (e, f), surgery (g, h), radiation (i, j), and chemotherapy (k, l).

**Figure 6:** 3- and 5-year receiver operating characteristic curves (ROC) of the validation group when predicting the OS (a) and CSS (b); 3- and 5-year calibration curves of the validation group when predicting the OS (c) and CSS (d).

**Table 1:** Characteristics of 1643 patients suffered penile cancer in SEER^1^ database.

Factors	Total	%	Development group	%	Validation group	%
Age						
50	176	10.7	126	10.9	50	10.2
50-59	272	16.6	180	15.6	92	18.7
60-69	418	25.4	291	25.3	127	25.8
70-79	413	25.1	300	26.1	113	22.9
80	364	22.2	254	22.1	110	22.4
Race						
Black	167	10.2	123	10.7	44	9.0
White	1393	84.8	965	83.8	428	87.0
Others^2^	83	5.0	63	5.5	20	4.0
Marital_status						
Never married	315	19.2	227	19.7	88	17.9
Single^3^	345	21.0	238	20.7	107	21.7
Married	983	59.8	686	59.6	297	60.4
Stage_T						
Stage_Tx	40	2.4	34	3.0	6	1.2
Stage_T1a	427	26.1	292	25.4	135	27.4
Stage_T1b	153	9.3	110	9.5	43	8.7
Stage_T1NOS	331	20.1	227	19.7	104	21.1
Stage_T2	380	23.1	270	23.4	110	22.4
Stage_T3	269	16.4	184	16.0	85	17.3
Stage_T4	43	2.6	34	3.0	9	1.9
Stage_N						
Stage_Nx	59	3.6	44	3.8	15	3.0
Stage_N0	1276	77.6	889	77.2	387	78.7
Stage_N1	92	5.6	61	5.3	31	6.3
Stage_N2	103	6.3	70	6.1	33	6.7
Stage_N3	113	6.9	87	7.6	26	5.3
Stage_M						
Stage_M0	1584	96.4	1117	97.0	467	94.9
Stage_M1	59	3.6	34	3.0	25	5.1
Primary_site						
Penis NOS	745	45.3	527	45.8	218	44.3
Prepuce	191	11.6	132	11.5	59	12.0
Glans	543	33.1	378	32.8	165	33.5
Body	88	5.4	58	5.0	30	6.1
Overlapping	76	4.6	56	4.9	20	4.1
Surgery^4^						
No	133	8.1	90	7.8	43	8.7
Destruction^5^	8	0.5	5	0.4	3	0.6
Excision^6^	454	27.6	315	27.4	139	28.3
Partial remove^7^	802	48.8	558	48.6	244	49.6
Total remove^8^	190	11.6	137	11.9	53	10.8
Radical surgery	52	3.2	42	3.6	10	2.0
Debulking surgery	4	0.2	4	0.3	0	0.0
Surgery_LN^9^						
No	1320	80.3	923	80.2	397	80.7
1-3	51	3.1	37	3.2	14	2.8
4	272	16.6	191	16.6	81	16.5
Radiation						
No	1532	93.3	1071	93.0	461	93.7
Before^10^	4	0.2	2	0.2	2	0.4
After^11^	107	6.5	78	6.8	29	5.9
Chemotherapy						
No	1445	87.9	1010	87.7	435	88.4
Yes	198	12.1	141	12.3	57	11.6
Histologic_type^12^						
805^13^	74	4.5	55	4.8	19	3.9
807^14^	1522	92.6	1062	92.2	460	93.5
808^15^	47	2.9	34	3.0	13	2.6
Endpoint						
Death	636	38.7	456	39.6	180	36.6
Cancer-specific death	250	15.2	175	15.2	75	15.2

^1^The Surveillance, Epidemiology, and End Results Program; ^2^includes patients whose race were not black or white; ^3^includes patients who are divorced, separated, windowed, and unmarried but have domestic partner; ^4^the surgery of the primary tumor; ^5^local tumor destruction, includes electrocautery, fulguration, or laser; ^6^local tumor excision, includes excisional biopsy, electrocautery, cryosurgery, and laser ablation; ^7^simple/partial surgical removal of primary site; ^8^total surgical removal of primary site (enucleation); ^9^number of lymph nodes removed in surgery; ^10^radiation before surgery; ^11^radiation after surgery; ^12^based on the 3rd Edition (ICD-O-3); ^13^includes verrucous papilloma, verrucous carcinoma, squamous cell papilloma, and papillary squamous cell carcinoma (8051, 8052); ^14^includes squamous cell carcinomas (8070-8076); ^15^includes Bowen disease, basaloid squamous cell carcinoma, and squamous cell carcinoma (clear cell type) (8081, 8083, 8084).

**Table 2:** Univariate and multivariate Cox analyses for OS based on penile cancer patients in development group.

Factors	Univariate analyses				Multivariate analyses			
	HR^1^	Lower.95	Upper.95	*P* value	HR^1^	Lower.95	Upper.95	*P* value
Age (<50 reference)								
50-59	1.131	0.7215	1.773	0.59124	1.2309	0.77595	1.9526	0.377541
60-69	1.090	0.7180	1.655	0.68520	1.1515	0.74684	1.7755	0.523055
70-79	1.802	1.2101	2.682	0.00374^∗∗^	2.0864	1.36742	3.1835	0.000646^∗∗∗^
80	3.385	2.2930	4.998	8.5*e*-10^∗∗∗^	4.1810	2.74884	6.3592	2.30*e*-11^∗∗∗^
Race (black reference)								
White	0.8057	0.6070	1.069	0.135	0.6494	0.48414	0.8710	0.003951^∗∗^
Others^2^	0.9103	0.5775	1.435	0.686	0.7800	0.49029	1.2408	0.294074
Marital_status (never married reference)								
Single^3^	1.1864	0.9044	1.5563	0.2172	0.9785	0.72886	1.3136	0.884948
Married	0.7774	0.6134	0.9853	0.0373^∗^	0.7197	0.55844	0.9277	0.011084^∗^
Stage_T (stage_Tx reference)								
Stage_T1a	0.4684	0.2733	0.8028	0.00579^∗∗^	0.9467	0.50694	1.7678	0.863414
Stage_T1b	0.7320	0.4115	1.3021	0.28843	1.3309	0.69430	2.5513	0.389203
Stage_T1NOS	0.5549	0.3230	0.9533	0.03290^∗^	1.0067	0.54747	1.8513	0.982764
Stage_T2	0.9758	0.5803	1.6410	0.92645	1.6022	0.88046	2.9156	0.122783
Stage_T3	1.2333	0.7278	2.0900	0.43589	1.8114	0.98363	3.3358	0.056522
Stage_T4	1.5350	0.7892	2.9854	0.20673	1.8733	0.91141	3.8505	0.087707
Stage_N (stage_Nx reference)								
Stage_N0	0.5758	0.3700	0.8961	0.0144^∗^	0.6480	0.40608	1.0340	0.068828
Stage_N1	1.0894	0.6282	1.8894	0.7604	1.1236	0.61476	2.0535	0.704932
Stage_N2	1.1808	0.6910	2.0179	0.5432	1.2421	0.68519	2.2515	0.475057
Stage_N3	1.7021	1.0337	2.8025	0.0366^∗^	1.9072	1.05862	3.4359	0.031585^∗^
Stage_M (stage_M0 reference)								
Stage_M1	5.657	3.866	8.277	<2*e*-16^∗∗∗^	2.9853	1.91073	4.6643	1.56*e*-06^∗∗∗^
Primary_site (penis NOS reference)								
Prepuce	0.7669	0.5524	1.065	0.1127	1.1000	0.77691	1.5574	0.591123
Glans	1.0115	0.8204	1.247	0.9144	0.8498	0.67695	1.0668	0.160644
Body	1.0510	0.6889	1.604	0.8175	1.0123	0.65225	1.5710	0.956641
Overlapping	1.4272	0.9619	2.117	0.0772	1.3770	0.91872	2.0640	0.121289
Surgery^4^ (no reference)								
Destruction^5^	0.2747	0.03796	1.9883	0.200768	0.3340	0.04502	2.4780	0.283505
Excision^6^	0.3556	0.25177	0.5022	4.33*e*-09^∗∗∗^	0.5427	0.35817	0.8224	0.003950^∗∗^
Partial remove^7^	0.5500	0.40583	0.7455	0.000117^∗∗∗^	0.6131	0.42087	0.8932	0.010823^∗^
Total remove^8^	0.7106	0.49235	1.0255	0.067942	0.8759	0.56608	1.3553	0.551899
Radical surgery	1.0104	0.62177	1.6418	0.966832	1.0677	0.61896	1.8419	0.813741
Debulking surgery	0.2530	0.03495	1.8317	0.173608	0.3071	0.04116	2.2910	0.249534
Surgery_LN^9^ (no reference)								
1-3	1.500	0.9563	2.353	0.0775	0.8601	0.51722	1.4302	0.561268
4	0.827	0.6365	1.075	0.1552	0.4983	0.36023	0.6894	2.60*e*-05^∗∗∗^
Radiation (no reference)								
Before^10^	2.909	0.7247	11.678	0.132	2.9055	0.70840	11.9172	0.138551
After^11^	1.502	1.0857	2.078	0.014^∗^	0.9870	0.67399	1.4455	0.946604
Chemotherapy (no reference)								
Yes	1.507	1.166	1.947	0.00174^∗∗^	1.0211	0.73072	1.4268	0.902703
Histologic_type^12^ (no reference)								
807^13^	2.412	1.326	4.389	0.00394^∗∗^	2.1134	1.14950	3.8854	0.016022^∗^
808^14^	2.701	1.240	5.883	0.01236^∗^	2.6931	1.21494	5.9697	0.014713^∗^

Signif. codes: 0 “^∗∗∗^” 0.001 “^∗∗^” 0.01 “^∗^” 0.05 “.” 0.1 “ ” 1. ^1^Hazard ratio; ^2^included patients who were not black or white; ^3^includes patients who are divorced, separated, windowed, and unmarried but have domestic partner; ^4^the surgery of the primary tumor; ^5^local tumor destruction, includes electrocautery, fulguration, or laser; ^6^local tumor excision, includes excisional biopsy, electrocautery, cryosurgery, and laser ablation; ^7^simple/partial surgical removal of primary site; ^8^total surgical removal of primary site (enucleation); ^9^number of lymph nodes removed in surgery; ^10^radiation before surgery; ^11^radiation after surgery; ^12^based on the 3rd Edition (ICD-O-3); ^13^includes squamous cell carcinomas (8070-8076); ^14^includes Bowen disease, basaloid squamous cell carcinoma, and squamous cell carcinoma (clear cell type) (8081, 8083, 8084).

**Table 3:** Univariate and multivariate Cox analyses for CSS based on penile cancer patients in development group.

Factors	Univariate analyses				Multivariate analyses			
	HR^1^	Lower.95	Upper.95	*P* value	HR^1^	Lower.95	Upper.95	*P* value
Age (<50 reference)								
50-59	0.8476	0.4903	1.465	0.554	0.8811	0.49409	1.5713	0.668058
60-69	0.7652	0.4621	1.267	0.299	0.7978	0.46209	1.3774	0.417553
70-79	0.7827	0.4717	1.299	0.343	1.029	0.58620	1.8046	0.921902
80	0.9276	0.5495	1.566	0.778	1.429	0.79779	2.5583	0.230137
Race (black reference)								
White	0.8822	0.5529	1.408	0.599	0.7507	0.45865	1.2287	0.254011
Others^2^	0.7126	0.3139	1.618	0.418	0.5988	0.25787	1.3906	0.232906
Marital_status (never married reference)								
Single^3^	0.7441	0.4810	1.1512	0.18431	0.7858	0.47988	1.2868	0.338117
Married	0.6157	0.4324	0.8767	0.00714^∗∗^	0.6577	0.44485	0.9724	0.035695^∗^
Stage_T (stage_Tx reference)								
Stage_T1a	0.2181	0.10326	0.4606	6.55*e*-05^∗∗∗^	0.7957	0.31850	1.9879	0.624708
Stage_T1b	0.4171	0.18737	0.9286	0.0322^∗^	1.151	0.44511	2.9769	0.771597
Stage_T1NOS	0.1487	0.06422	0.3442	8.56*e*-06^∗∗∗^	0.4869	0.18971	1.2497	0.134547
Stage_T2	0.5935	0.30062	1.1717	0.1328	1.175	0.50536	2.7308	0.708256
Stage_T3	1.0107	0.51361	1.9887	0.9755	1.530	0.65305	3.5829	0.327708
Stage_T4	1.9844	0.89128	4.4184	0.0933	2.175	0.87897	5.3800	0.092794
Stage_N (stage_Nx reference)								
Stage_N0	0.2941	0.1568	0.5517	0.000138^∗∗∗^	0.3897	0.19447	0.7808	0.007870^∗∗^
Stage_N1	0.9554	0.4387	2.0807	0.908571	0.7665	0.31698	1.8533	0.554915
Stage_N2	1.4215	0.6961	2.9028	0.334280	0.9938	0.43808	2.2543	0.988048
Stage_N3	2.2364	1.1506	4.3469	0.017615^∗^	1.575	0.71318	3.4777	0.261155
Stage_M (stage_M0 reference)								
Stage_M1	11.5	7.289	18.13	<2*e*-16^∗∗∗^	2.72	1.57625	4.6935	0.000325^∗∗∗^
Primary_site (penis NOS reference)								
Prepuce	0.4812	0.2491	0.9296	0.0295^∗^	1.036	0.51798	2.0727	0.920041
Glans	1.2063	0.8702	1.6722	0.2604	1.026	0.71082	1.4806	0.891476
Body	1.0869	0.5452	2.1672	0.8128	0.918	0.44012	1.9150	0.819678
Overlapping	1.4768	0.7853	2.7773	0.2263	1.375	0.70899	2.6685	0.345756
Surgery^4^ (no reference)								
Destruction^5^	0.4711	0.06416	3.4594	0.4594	1.149	0.14605	9.0462	0.894733
Excision^6^	0.0860	0.04387	0.1686	9.03*e*-13^∗∗∗^	0.2622	0.11916	0.5770	0.000879^∗∗∗^
Partial remove^7^	0.3971	0.26150	0.6029	1.46*e*-05^∗∗∗^	0.6501	0.36843	1.1472	0.137283
Total remove^8^	0.5274	0.31219	0.8910	0.0168^∗^	0.8146	0.42677	1.5549	0.534119
Radical surgery	0.9327	0.48473	1.7946	0.8346	1.326*e*	0.61167	2.8763	0.474444
Debulking surgery	0.4784	0.06511	3.5149	0.4687	0.3596	0.04589	2.8182	0.330242
Surgery_LN^9^ (no reference)								
1-3	3.219	1.8514	5.596	3.43*e*-05^∗∗∗^	1.326*e*+00	0.68914	2.5514	0.398109
4	1.438	0.9993	2.069	0.0504	6.195*e*-01	0.39521	0.9712	0.036836^∗^
Radiation (no reference)								
Before^10^	2.264*e*-06	0.000	Inf	0.992236	6.685*e*-06	0.00000	Inf	0.992907
After^11^	2.364	1.525	3.666	0.000121^∗∗∗^	7.886*e*-01	0.46332	1.3421	0.381292
Chemotherapy (no reference)								
Yes	3.704	2.686	5.108	1.41*e*-15^∗∗∗^	1.525*e*+00	0.98840	2.3538	0.056489
Histologic_type^12^ (no reference)								
807^13^	3.343	1.0673	10.47	0.0383^∗^	2.655*e*+00	0.81747	8.6243	0.104237
808^14^	3.749	0.9373	15.00	0.0617	4.403*e*+00	1.04301	18.5875	0.043667^∗^

Signif. codes: 0 “^∗∗∗^” 0.001 “^∗∗^” 0.01 “^∗^” 0.05 “.” 0.1 “”. 1; Inf: infinity. ^1^Hazard ratio; ^2^included patients who were not black or white; ^3^includes patients who are divorced, separated, windowed, and unmarried but have domestic partner; ^4^the surgery of the primary tumor; ^5^local tumor destruction, includes electrocautery, fulguration, or laser; ^6^local tumor excision, includes excisional biopsy, electrocautery, cryosurgery, and laser ablation; ^7^simple/partial surgical removal of primary site; ^8^total surgical removal of primary site (enucleation); ^9^number of lymph nodes removed in surgery; ^10^radiation before surgery; ^11^radiation after surgery; ^12^based on the 3rd Edition (ICD-O-3); ^13^includes squamous cell carcinomas (8070-8076); ^14^includes Bowen disease, basaloid squamous cell carcinoma, and squamous cell carcinoma (clear cell type) (8081, 8083, 8084).

## Data Availability

The dataset supporting the conclusions of this study is available in the SEER database.
